The article "Identification of Good Practices in Long-Term Exercise-Based Rehabilitation Programs in Stroke Patients" was published in 2021. Journal: Biomed Res Int.

# Identification of Good Practices in Long-Term Exercise-Based Rehabilitation Programs in Stroke Patients

**DOI:** 10.1155/2021/9202716

**Published:** 2021-09-27

**Authors:** Dimitra Mameletzi, Maria Anifanti, Kristina Baotić, Andrea Bernetti, Hrvoje Budinčević, Petra Črnac Žuna, Asterios Deligiannis, Zekie Dennehy, Andrea Ferrari, Dolores Forgione, Jurlina Hrvoje, Maura Ilardi, Borbála Sára Kiss-Szemán, Nikolaos Koutlianos, Iveta Kovářová, Massimiliano Mangone, Marco Paoloni, Lolita Rapolienė, Artūras Razbadauskas, Aelita Skarbalienė, Egidijus Skarbalius, Evangelia Kouidi

**Affiliations:** ^1^Laboratory of Sports Medicine, Aristotle University of Thessaloniki, Greece; ^2^Croatian Stroke Society, Croatia; ^3^Department of Physical Medicine and Rehabilitation, Sveti Duh University Hospital, Zagreb, Croatia; ^4^Department of Anatomical, Histological, Legal and Locomotor Sciences of Sapienza University, Italy; ^5^Department of Neurology, Stroke and Intensive Care Unit, Sveti Duh University Hospital, Zagreb, Croatia; ^6^Faculty of Medicine, University J.J. Strossmayer, Osijek, Croatia; ^7^CEREBRUM-Association of People with Acquired Brain Injuries and their Families, Czech Republic; ^8^Istituto Europeo per lo Sviluppo Socio Economico (ISES), Italy; ^9^Dom zdravlja Zagrebačke županije, Velika Gorica, Croatia; ^10^Klaipėda University, Lithuania

## Abstract

Physical activity is an important factor for primary and secondary stroke prevention. The process of stroke rehabilitation includes early and late physical activity and exercise, which prevents further stoke and improve patients' quality of life. MY WAY project, an ERASMUS+ SPORT program, is aimed at analyzing and developing or transferring best innovative practices related to physical activity and exercise enhancing health in poststroke patients. The aim of the study was to identify, analyze, and present the good practices and strategies to encourage participation in sport and physical activity and engage and motivate chronic stroke patients to perform physical activity changing their lifestyle and to maintain a high adherence to long-term exercise-based rehabilitation programs. Our results demonstrated that unified European stroke long-term exercise-based rehabilitation guidelines do not exist. It seems that low training frequency with high aerobic exercise intensity may be optimal for improved physical performance and quality of life in combination with a high adherence. It is important to optimize the training protocols suitable for each patient. The continuous education and training of the specialized professionals in this field and the presence of adequate structures and cooperation between different healthcare centers are important contributors. The clear objective for each country should be to systematically make the necessary steps to enhance overall exercise-based stroke rehabilitation attendance in the long term. Long-term interventions to support the importance of physical exercise and lifelong exercise-based rehabilitation in chronic stroke patients should be created, what coincides with the goal of the MY WAY project.

The article "Identification of Good Practices in Long-Term Exercise-Based Rehabilitation Programs in Stroke Patients" was published in 2021. Journal: Biomed Res Int.

## 1. Introduction

Due to the aging of the population and the increased prevalence of chronic diseases, such as diabetes mellitus, hyperlipidemia, and hypertension, there is a significant rise in stroke incidence among European countries and worldwide, during the last decades [1, 2]. Together with the welcome improvement in the survival rates, the number of people who have had a stroke and must live with its consequences needing specialist supportive care and rehabilitation is increased [3, 4]. Stroke survivors can experience a wide range of negative physical and mental consequences that are long lasting, including problems with mobility, vision, speech, and memory; personality changes; cognitive impairments; fatigue; and depression. Poststroke problems affect patients' ability to complete daily activities at home and to participate in the community [5].

An effective health care planning and adequate resource allocation across Europe is needed to deal with the rising number of people living with the long-term effects of stroke. In particular, access to rehabilitation therapy, mainly postacute care, must be improved. The hope is that in Europe everyone gets the long-term support they need to regain as much independence as possible.

Long-term exercise-based rehabilitation is aimed at enabling people with disabilities to reach and maintain optimal physical, intellectual, psychological, and/or social function. European stroke care guidelines make recommendations for the elements of rehabilitation [6], although there is not enough evidence to ensure the exact content of the recommended therapies. Additionally, there is no uniform approach in the EU and no common exercise-based stroke rehabilitation protocol is suggested among the European countries [7, 8]. Nevertheless, physical activity and exercise are highly recommended in the chronic phase to sustain functions gained in rehabilitation and as part of long-term secondary prevention to reduce the risk of recurrent stroke and other vascular events [9, 10].

Research suggests that stroke patients may benefit from early exercise training aiming to enhance their exercise capacity, help prevent further strokes, and improve patients' quality of life [11, 12]. It seems that exercise training has multiple mechanisms of action. Several studies have shown that exercise training could protect the brain from stroke injury by mechanisms involved in the regulation of cerebral edema, cellapoptosis, oxidative injury, and stem cell [13]. In addition, it has been demonstrated that exercise facilitates neuroplasticity by promoting the compensation of surviving brain areas; improving interhemispheric connections; increasing synaptic plasticity through regulating neurotrophins, synaptic activity, and structure; and accelerating neuronal reorganization and regeneration [14]. A systematic review evidence showed that exercise interventions are beneficial for patients with a number of conditions that are comorbid conditions or risk factors for stroke, by improving vascular risk factors in obesity and type II diabetes, reducing blood pressure, and improving cardiovascular mortality and depressive symptoms [12]. Hence, development of new interventions is needed to help stroke survivors achieve a more active lifestyle to maintain the functional levels achieved during stroke unit treatment and early poststroke rehabilitation [15]. MY WAY project, which is an ERASMUS+ SPORT program that involves experts from Croatia, Czech Republic, Greece, Italy, and Lithuania, is aimed at covering this gap. MY WAY project seeks to develop, implement, and transfer innovative practices related to physical activity and exercise enhancing health in poststroke patients. To achieve this goal, the identification of good practices in the field of long-term exercise-based rehabilitation is important. The aim of the present study was to identify, analyze, and present the good practices and strategies to encourage participation in sport and physical activity and engage and motivate chronic stroke patients to perform physical activity changing their lifestyle and to maintain a high adherence to long-term exercise-based rehabilitation programs.

The article "Identification of Good Practices in Long-Term Exercise-Based Rehabilitation Programs in Stroke Patients" was published in 2021. Journal: Biomed Res Int.

## 2. Methodology

Innovative practices have been collected through literature review of international publication databases and directly from partner countries through their own research. Each partner identified good practices in the project field, exploring exercise-based interventions and promoting and inhibiting factors of physical activity and exercise in stroke patients, through a wide literature review of international publication databases. Moreover, an analysis of successful and unsuccessful local experiences was performed to find for the different European local contexts cost-effective and applicable solutions.

The collection and analysis of good practices have been performed in three steps:

1. Interventions of international literature database origin have been surveyed through a detailed literature review
2. MY WAY project partners have been asked to assess these interventions along several indicators
3. MY WAY project partners have been asked to collect recent interventions from their own national context

### 2.1. Step 1: Literature Review

As a first step, toward identifying good practices in long-term exercise-based stroke rehabilitation, the MY WAY consortium performed a comprehensive literature review. After setting the research question, inclusion and eligibility criteria set the boundaries for the study review. White literature search through PubMed and free internet search were performed. The search strategy and plan were developed with some “search terms” (stroke, cerebrovascular accident +/- patients +/- country or region name + keyword or combination of keywords of interest; rehabilitation; physical activity; exercise; training; intervention; mobility; physical training; long-term rehabilitation; walking; balance; etc.) identified. During this process, the following set criteria were applied:

The sources for information needed to

- be randomized controlled trials published in peer-reviewed journal
- include a comprehensive evaluation system, preferably based on quantifiable results
- provide at least some basic information about intervention design, people involved, identified barriers, sustainability, and transferability and
- contain any innovative idea or element in the field of physical activity and exercise in stroke patients

### 2.2. Step 2: Assessment of the Exercised-Based Interventions

For each intervention, a set of features was also collected, such as date of intervention, country of intervention, intervention/control group size, gender mix, intervention length, assessment periods, outcome measures, and limitations. Then, a questionnaire has been prepared for MY WAY project partners to evaluate the selected interventions. The following four dimensions needed to be evaluated: relevance, quality, effectiveness, and sustainability. A weighted scoring system was introduced to obtain an objective evaluation system, each indicator summing up to 100 points.

Apart from analyzing the scores, a thorough examination of intervention texts and answers to elaborative questions were the basis of nonquantifiable insights. Qualitative and quantitative analyses together provide a wealth of conclusions from the interventions.

### 2.3. Step 3: EU Partners' Country Interventions

Each partner was asked to provide and analyze at least two published studies, indicative of the exercise-based interventions provided in patients after stroke in their EU country. As a priority, the main criterion was to include interventions related to long-term exercise-based poststroke rehabilitation programs. Furthermore, the intention was to include different kinds of exercise-based programs that constitute good practices related to physical activity/exercise/sports enhancing all aspects of health in poststroke patients. Partners were encouraged to choose and analyze randomized controlled trials published in peer-reviewed scientific journals. However, practical and concrete actions were also accepted. In addition, partners were asked to reveal the initiatives that could be useful in each country to increase stroke patients' effective participation in exercise activities.

The article "Identification of Good Practices in Long-Term Exercise-Based Rehabilitation Programs in Stroke Patients" was published in 2021. Journal: Biomed Res Int.

## 3. Results

### 3.1. Literature Review Analysis

During the first step analysis, according to the eligibility criteria, 30 publications with 30 exercise-based rehabilitation programs implemented in developed countries worldwide were identified. During the second stage analysis, thirteen randomized controlled trials with exercise-based interventions after stroke fulfilled the set criteria (Table 1). Publication dates of the selected 13 international interventions were between 2011 and 2020. The average publication year was 2017, while 12 interventions were recent (within five years). Thus, 65 assessments derived from the five MY WAY partners were collected. The assessments included the quantitative and qualitative analyses and evaluation of the 13 international exercise-based interventions, concerning relevance, quality, effectiveness, and sustainability.

#### 3.1.1. Relevance

The relevance of the interventions was evaluated by questions inquiring about the potential of the intervention to serve the needs of different target groups and their consequent success in this respect. Overall, the analyzed interventions have scored very well on the relevance scale. With a maximum score of 100, four of the examined interventions were over 75 points. Only one intervention was below 50 points (49 points to be exact).

The high scores were mainly due to the fact that the examined interventions were well planned and very recent, since the 12 out of 13 have been published after 2016 (only one was published in 2011). However, only three interventions came from an EU country (plus one from the UK). It was clear that many more European-based interventions would be needed to create more robust evidence in support of exercise-based rehabilitation in poststroke patients.

One of the most important aspects of the relevance-analysis was measuring the value provided to the target groups. According to the evaluations, it was clearly stated that the interventions served patient needs better and were more polarized in relation to patients.

The article "Identification of Good Practices in Long-Term Exercise-Based Rehabilitation Programs in Stroke Patients" was published in 2021. Journal: Biomed Res Int.

#### 3.1.2. Quality

The quality of an intervention was greatly affected by the number of involved participants. In this respect, the examined interventions performed rather poorly.

The number of participants was interpretable in all 13 interventions, and this was below 100 in 9 cases (even below 50 in 6 interventions), only two interventions having more than 300 participants, and precisely only one with more than 400 (408 to be exact). Low participant numbers had a mitigating effect on the strength of the interventions. The small group of participants in the studies provided a weak base for statistical analysis, and again, even more importantly, they may not be enough to grab the attention of the real decision makers, who were in position to act on the results and implement changes in the structure of stroke exercise-based rehabilitation.

With respect to the intervention length, only 5 out of the 13 studies spanned a time of at least three months and one of them only lasted for over a year (18 months to be exact). The only intervention (regular coaching to perform 30 min physical activity daily every day and 45-60 min of physical exercise with 2–3 bouts of vigorous intensity levels every week) lasting 18 months had significantly increased adherence to the intervention associated with improved cognitive function that shorter interventions could not have measured. Long interventions have the potential to alter perceptions of patients and medical professionals alike.

#### 3.1.3. Sustainability

An important factor to be considered was whether the positive effects of an intervention outlasted the project, providing future benefits even without further investment. Unfortunately, as the analyzed studies were trying to create controlled environments with limited desire for immediate practical application, sustainability was rarely considered an important factor. It was possible nevertheless in many cases to draw very plausible conclusions based on the information provided.

The question, ‘Would you recommend this intervention to be implemented on a larger scale?,' measured sustainability explicitly. An interesting finding was a relatively high disagreement with regards to the same interventions. The level of differences was demonstrated by Figure 1, showing the positive and the negative evaluations between the scores for each of the 13 interventions. Three interventions showed only positive answers, while all evaluators replied negatively only in one intervention.

*Τ*he sustainability results indicated that every country has its own long-term exercise-based rehabilitation settings, and it was difficult to implement new interventions in larger scale. A successful intervention in a particular setting did not guarantee similar results, in case that the stakeholders' perceptions were different. However, evaluators clearly agreed that the main stakeholders of stroke exercise-based rehabilitation interventions were patients and healthcare professionals.

The article "Identification of Good Practices in Long-Term Exercise-Based Rehabilitation Programs in Stroke Patients" was published in 2021. Journal: Biomed Res Int.

#### 3.1.4. Effectiveness

Effectiveness is the capability of producing a desired result. An intervention was considered effective when it had been evaluated, and the final results showed to have reached its target for specific indicators with a determined agreed tolerance.

Most of the included studies were from rehabilitation center members who had suffered stroke, and they enrolled more participants with hemorrhagic stroke. Eight out of the 13 studies included patients with first onset of stroke more than 6 months prior to participation.

The duration of all exercise interventions ranged from 20 to 90 minutes per session, 2 to 5 times per week for 4 to 12 week period (with the exception of one study lasting 18 months). The training programs involved aerobic training, strength training, and/or core stabilization and balance exercises (6, 2, and 5 studies, respectively). Four studies assessed the effects of mixed training (exercises on a vibrating platform and walking on a treadmill, dual-task walking program, virtual reality exercises with Wii Fit and Wii Balance board, and tailored training programs based on the patient's preferences and goals). The majority of the studies focused on land-based exercise (11 studies). Only 2 out of the 13 studies comprised aquatic training.

The effects of each exercise training mode have been assessed using a variety of questionnaires, impairment and balance scales, standardized cognitive function neuropsychological tests, and simple functional tests (activity monitors, dynamometry, mobility tests, the Modified Ashworth Scale, the Korean Trunk Impairment Scale, the 6-Minute Walk Test, the Balance Walking Speed Test, the Timed Up and Go Test, the Static Balance Index, the Berg Balance Scale, the Postural Assessment Scale for Stroke, the Functional Reach Test, the Barthel Index, the Postural Assessment Scale for Stroke Patients, the European Quality of Life Scale, the Stroke Impact Scale, the Fugl-Meyer Assessment of Motor Recovery in the legs, the Berg Balance Scale, the Activities-Specific Balance Confidence Scale, the Activities of Daily Living-Instrumental Activities of Daily Living Scale, and the Stroke Impact Scale).

All included trials indicated that exercise training had a positive impact on physical and/or cognitive functions. The majority of the studies found that exercise training enhances walking performance and mobility (9 studies), as well as balance ability (7 studies). Three studies showed significant improvements in patients' health-related quality of life and motor recovery and two studies reported enhanced trunk control and performance of activities of daily living. Finally, one study found that increased adherence to the physical activity intervention was associated with improved cognitive function. Details of the nature and dose of the exercise training intervention studies and their main outcomes are summarized and presented in Table 1.

The article "Identification of Good Practices in Long-Term Exercise-Based Rehabilitation Programs in Stroke Patients" was published in 2021. Journal: Biomed Res Int.

The extent to what the evaluators from the different partner countries agreed on the effectiveness of the different interventions has also been examined. Project partners were in almost complete agreement in the case of two interventions and the opinions on the rest were also quite similar. This result proved that professional views of effectiveness were much more uniform than that of sustainability. However, effectiveness scores showed the largest dispersion of all indicator categories (Figure 2). Average relevance and sustainability scores were markedly lower compared to effectiveness and quality scores.

### 3.2. Analysis of the Partners' Countries Interventions

Ten long-term exercise-based stroke rehabilitation-related interventions have been collected from the partner countries, two from each partner (Table 2). There were no preconditions attached to these interventions, and consequently, they were very much varied. Most of the interventions were scientific studies, while others were practical and concrete actions.

The two Croatian interventions used individualized approaches to minimize barriers and side effects and to increase patients' motivation [16, 17]. The two Czech studies concerned the use of novel robotic techniques to improve outcomes and patients' motivation [18, 19]. The two Greek studies are aimed at detecting the effectiveness of different modalities of interventions, in order to improve the quality of rehabilitation interventions [20, 21]. The two Italian studies evaluated the effectiveness, in both the short and long period of therapeutic patient education, and adapted physical activity intervention in stroke survivors [22] and addressed the crucial issue of intensity that the exercise-based rehabilitation programs of stroke patients should have [23]. Finally, the two Lithuanian interventions were both offered in the Palanga Rehabilitation Hospital and used novel techniques to enhance motivation of the patients (not published interventions, Palanga Rehabilitation Hospital, 2020).

The main characteristics of the strategies collected from the partners' countries' interventions aiming to increase participation in long-term exercise-based stroke rehabilitation activities and improve the efficiency of a comprehensive long-term poststroke rehabilitation system are summarized in Table 3.

The article "Identification of Good Practices in Long-Term Exercise-Based Rehabilitation Programs in Stroke Patients" was published in 2021. Journal: Biomed Res Int.

## 4. Discussion

The results of the present study demonstrated that unified European chronic stroke long-term exercise-based rehabilitation guidelines do not exist. Though evidence supports that secondary and tertiary preventions have the biggest impact on health, apparently few interventions are performed. Although the European Stroke Organization (ESO) has already formulated rehabilitation recommendations, these are not widely practiced in the EU Member States [6]. This fact itself should be more than alarming to stakeholders to start designing interventions and studies aiming to promote long-term exercise-based chronic stroke rehabilitation programs. There is a trend in global health care, exercise-based rehabilitation becoming more popular that will hopefully have a positive effect on the number and quality of initiatives aimed at improving current long-term exercise-based programs. The MY WAY project fits well into this emerging trend.

Concerning the common characteristics of the interventions with regards to relevance, it seemed that walking and balance were important functions to recover after stroke and functional limitations frequently necessitated ongoing exercise-based rehabilitation [24–27]. Since trunk muscle weakness in chronic stroke patients was related to poor balance and mobility-related functional activities, strengthening the trunk muscles led to improvement in activities of daily living, including trunk performance and balance [28, 29]. Therefore, interventions that could alleviate balance impairments and improve balance and functional mobility should be important goals of long-term exercise-based rehabilitation [30–32]. In addition, group activities provided social support and participation, which improved or preserved the quality of life [32].

As for the common characteristics of the interventions with regards to quality, the low participation rate in the interventions reduced the quality and the relevance of each intervention as well as the accuracy of the results. It is important to optimize the training protocols suitable for each patient. Early initiation, assessment of each patient's functional limitation, and the application of long-term, specific, and intensive exercise-based rehabilitation programs are recommended for more benefits [33–35]. Moreover, common issues identified in many interventions is the small sample size, the lack of or short follow-up assessments, and the limited types of stroke studied (usually mild-to-moderate). The introduction of many large-scale interventions is required.

The article "Identification of Good Practices in Long-Term Exercise-Based Rehabilitation Programs in Stroke Patients" was published in 2021. Journal: Biomed Res Int.

Furthermore, it seems that low training frequency with high aerobic exercise intensity may be optimal for improved physical performance and quality of life in combination with a high adherence. The outcomes of the exercise rehabilitation programs in stroke patients persisted at 6-month follow-up, especially in patients with an interest in training [26]. In addition, since chronic stroke rehabilitation often requires multiple behavior modifications, health education provided to all individuals throughout the intervention period contributes to this direction [32].

Concerning sustainability, tailored training programs, based on the patient's preferences and goals, are suggested [30, 32, 35]. Moreover, a series of measures, including small group sizes, community health centers near the subjects, weekly telephone follow-ups and monthly family follow-ups, group training, stratification into subgroups based on stroke severity and supposed reversibility, and health education should be taken to ensure the adherence and safety of chronic stroke patients participating in physical activity and exercise training programs [32, 34, 35].

Regarding effectiveness, it seems that increased adherence to physical activity and exercise is associated with improved functional capacity and cognitive function, indicating that the intervention dose might be of importance to achieve a benefit [33, 35]. In addition, while light-to-moderate physical activity could have a beneficial effect on cognitive flexibility and brain reserve, an effect through neurogenesis and angiogenesis may be achieved through interventions with higher intensities [35]. Furthermore, aerobic physical fitness, hydrotherapy, and Wii Fit-based balance training programs should be considered effective tools for improving postural balance and mobility in chronic stroke patients [27, 31, 36].

One main goal of the MY WAY project was to identify interventions that could be effective once introduced in real life, in the partner countries. An important part of this strategy was to reveal current situation and identify proved good practices and strategies to increase the efficiency of chronic stroke rehabilitation practices. To identify good examples of long-term exercise-based chronic stroke rehabilitation, MY WAY project partners collected recent interventions from their own national context.

The first Croatian intervention (stationary vs. home rehabilitation) showed that an individual approach to every stroke patient, with the evaluation of risk factors, comorbidities, socioeconomic situation, age, and gender, would enable the most appropriate rehabilitation modality with the best cost-effectiveness [16]. The second Croatian intervention (rehabilitation with mirror-induced visual illusion) highlighted the efficacy of mirror therapy in the improvement of motor function in the upper limb in poststroke patients, leading to a greater potential of self-care and activities of daily living [17].

The article "Identification of Good Practices in Long-Term Exercise-Based Rehabilitation Programs in Stroke Patients" was published in 2021. Journal: Biomed Res Int.

The Czech robotic rehabilitation study concluded that robotic technologies, providing optimal repeated rehabilitation stretching of spastic muscles can be used as supplement or substitution of the stretching techniques [18]. In another Czech study, where Amadeo instrument was used, the robotic assisted hand treatment of patients in the chronic phase after brain vascular event was evaluated very positively by the patients [19]. Thus, the use of novel robotic techniques developed over the last decade provides the perspective of improving results of rehabilitation, as they proved useful for increasing the motor activity output.

Additionally, cervical isometric exercises were shown to be beneficial in helping patients improve their cervical spine alignment and overcome deglutition disorders [20]. Another Greek study showed that the music-based exercise programs had a positive effect on mood profile and recovery rate in stroke patients [21].

The “adaptive physical activity with therapeutic patient education” Italian study observed a significant improvement on mobility, balance, and on patients' perception of recovery from the acute phase [22]. The increased number of participants showed the value of a large sample exercise-based rehabilitation studies; moreover, the contribution of a long-term follow-up (12 months) showed the importance to verify the intervention long-term effects. Overall, adapted physical activities associated to therapeutic patient education were identified as a useful and potentially cost-effective intervention to maintain and improve activities of daily living, reduce fractures, and recourse to rehabilitation treatments [22]. The Italian “low intensity endurance and resistance training” study addressed the crucial issue of intensity that the exercise-based rehabilitation programs of stroke patients should have. It was shown that an 8-week, community-based, progressive mixed endurance-resistance exercise program at lower cardiovascular and muscular load leads to better mobility benefits than a higher-intensity program in chronic stroke survivors [23].

The “virtual reality and traditional physiotherapy” Lithuanian study revealed that the application of a PC virtual reality system enhanced rehabilitation in stroke patients (unpublished intervention, Palanga Rehabilitation Hospital, 2020). Specifically, it was shown that patients who spent the most time on virtual reality therapy procedures during their departure from the rehabilitation center significantly improved their independence. In order to maintain such motivation for a longer period, it is recommended to train continuously and expand the computer package with new programs. Furthermore, virtual reality seems to be a useful way to involve patients in the long-term exercise-based rehabilitation process [37]. The second Lithuanian study (gait training with KinisiForo System) showed that after gait training with novel exercise technologies, patients experience higher improvements in gait speed (unpublished intervention, Palanga Rehabilitation Hospital, 2019) [37].

The article "Identification of Good Practices in Long-Term Exercise-Based Rehabilitation Programs in Stroke Patients" was published in 2021. Journal: Biomed Res Int.

Synthesizing the evidence on facilitators and barriers to the effective implementation of exercise-based rehabilitation programs, the main factor that positively influences the sustainability and transferability of the interventions is the cooperation between specialist doctors, dedicated professionals, and patients. Additionally, the continuous education and training of the specialized professionals in this field, the presence of adequate structures and cooperation between different healthcare centers are important contributors. On the other hand, the main aspects that negatively affect sustainability and transferability are the potential difficulty among different regions to obtain funds in the public healthcare system to guarantee an adequate delivery of the program, the lack of a structured and organized regional healthcare network, and the reduced advertising promotion of relevant projects. The clear objective for each country should be to systematically make the necessary steps to enhance overall exercise-based stroke rehabilitation attendance in the long term.

## 5. Conclusion

In conclusion, the analysis of good practices explored promoting and inhibiting factors of physical activity and exercise in chronic stroke patients. Long-term interventions to support the importance of physical exercise and lifelong exercise-based rehabilitation in chronic stroke patients should be created. The MY WAY goal is that every stroke patient gets the long-term support he/she needs to regain as much independence as possible and to improve his/her quality of life [37].

## Figures and Tables

**Figure 1:** Sustainability evaluations of the 13 interventions.

**Figure 2:** Box plot of the indicator-specific distribution of the interventions.

**Table 1:** Overview of the 13 randomized controlled trials including exercise-based interventions after stroke.

Study	Participants	Intervention	Main findings
Aguiar et al., 2018 [33]	22 adults with chronic stroke	Experimental group: aerobic treadmill training at 60–80% of heart rate reserve. Control group: outdoor-overground walking below 40% of heart rate reserve. Both groups: three 40 min sessions/week over 12 weeks	Aerobic treadmill training improved quality of life. Aerobic treadmill training or outdoor-overground walking improved depression, endurance, and mobility

Choi et al., 2017 [24]	30 ambulatory chronic stroke patients allocated to whole-body vibration combined with treadmill training (WBV-TT) group or treadmill training (TT) group	The WBV-TT group performed 6 types of exercises on a vibrating platform for 4.5 minutes and then walked on the treadmill for 20 minutes. The TT group conducted the same exercise on a platform without vibration and then walked on the treadmill in the same manner. The vibration lasted for 45 seconds in each exercise, and the intervention was performed 3 times weekly for 6 weeks. The treadmill walking speed was gradually increased by 5% in both groups.	The WBV-TT group showed significant improvements in walking performance with respect to walking speed, cadence, step length, stride length, single-limb support, double-limb support, and 6-minute walk test compared with baseline (*p* < 0.05). Significant improvements were also seen in walking speed, step length, stride length, and double-limb support compared with the TT group (*p* < 0.05)

Duncan et al., 2011 [30]	408 participants who had had a stroke 2 months earlier according to the extent of walking impairment—moderate (able to walk 0.4 to <0.8 m per second) or severe (able to walk <0.4 m per second)—and randomly assigned them to one of three training groups	One group received training on a treadmill with the use of bodyweight support 2 months after the stroke had occurred (early locomotor training), the second group received this training 6 months after the stroke had occurred (late locomotor training), and the third group participated in an exercise program at home managed by a physical therapist 2 months after the stroke (home exercise program). Each intervention included 36 sessions of 90 minutes each for 12 to 16 weeks	All groups had similar improvements in walking speed, motor recovery, balance, functional status, and quality of life

Ehrensberger et al., 2019 [34]	32 patients with chronic stroke	A 4 wk isometric strength training program performed with the less-affected upper limb three times per week. Participants in the mirror and strength training group observed the reflection of the exercising arm in the mirror. Participants in the strength training only group exercised without a mirror entirely	Self-perceived impact of stroke improved. The feasibility and potential effectiveness of mirror-aided cross-education compared with cross-education only for upper limb motor recovery were established

Haruyama et al., 2017 [28]	32 participants randomly assigned to an experimental group or a control group (*n* = 16 each)	The experimental group received 400 minutes of core stability training in place of conventional programs within total training time (20 minutes of core stabilization exercises within each daily training session, 5 times a week, for 4 weeks), while the control group received only conventional programs	Beneficial effects on trunk function, standing balance, and mobility

Ihle-Hansen et al., 2019 [35]	362 patients with first ever or recurrent stroke due to infarction and intracerebral hemorrhage	The intervention group received individualized coaching for physical activity 30 min daily, and 45–60 min physical exercise including 2–3 bouts of vigorous activity every week	Positive association between increasing adherence to the intervention and cognitive function

Karasu et al., 2018 [31]	23 subacute and chronic stroke patients were randomly assigned to either the experimental group (*n* = 12) or the control group (*n* = 11)	Both groups participated in conventional balance rehabilitation exercises, 2–3 h a day, 5 days a week. The experimental group received 20 sessions of 20 min of balance exercise, 5 days a week, for 4 consecutive weeks, with Wii Fit and Wii Balance board, in addition to conventional rehabilitation	Wii Fit-based balance rehabilitation could represent a useful adjunctive therapy to traditional treatment to improve static and dynamic balance, functional motor ability, and independence in stroke patients

Nave et al., 2019 [36]	200 adults with subacute stroke (days 5-45 after stroke) with a median National Institutes of Health stroke scale (NIHSS, range 0-42 points, higher values indicating more severe strokes) score of 8 (interquartile range 5-12) were randomly assigned (1 : 1) to aerobic physical fitness training (*n* = 105) or relaxation sessions (*n* = 95, control group) in addition to standard care	Participants received either aerobic, bodyweight supported, treadmill-based physical fitness training or relaxation sessions, each for 25 minutes, five times weekly for four weeks, in addition to standard rehabilitation therapy	Change in maximal walking speed in the 10 m walking test and change in Barthel index scores three months after stroke compared with baseline. Compared with relaxation, aerobic physical fitness training did not result in a significantly higher mean change in maximal walking speed (adjusted treatment effect 0.1 m/s (95% confidence interval 0.0 to 0.2 m/s), *p* = 0.23) or mean change in Barthel index score (0 (−5 to 5), *p* = 0.99) at three months after stroke

Pang et al., 2018 [25]	84 chronic stroke patients (24 women; age, 61.2 ± 6.4 years; time since stroke onset, 75.3 ± 64.9 months) with mild to moderate motor impairment (Chedoke-McMaster leg motor score: median, 5; interquartile range, 4–6) were randomly allocated to the dual-task balance/mobility training group, single-task balance/mobility group, or upperlimb exercise (control) group	Each group exercised for three 60-minute sessions per week for 8 weeks	The dual-task program was effective in improving dual-task mobility, reducing falls and fall-related injuries. It had no significant effect on activity participation or quality of life

Park et al., 2019 [29]	29 chronic stroke patients were randomly allocated to the land-based and aquatic trunk exercise group (*n* = 14) and control group (*n* = 15)	Land-based and aquatic trunk exercises (LATE) were performed for 30 minutes per day, 5 days per week, for 4 weeks as an adjunct to 30 minutes of conventional physical therapy. The control group underwent only conventional physical therapy for 30 minutes each time, twice per day, 5 days per week, for 4 weeks	The LATE program helped improve trunk control, balance, and activities of daily living

Sandberg et al., 2016 [26]	56 patients (28 women) who had a mild stroke (98% ischemic) and were discharged to independent living and enrolled 20 days (median) after stroke onset	60 minutes of group aerobic exercise, including 2 sets of 8 minutes of exercise with intensity up to exertion level 14 or 15 of 20 on the Borg rating of perceived exertion scale, twice weekly for 12 weeks (*n* = 29). The nonintervention group (*n* = 27) received no organized rehabilitation or scheduled physical exercise	Intensive aerobic exercise twice weekly improved aerobic capacity, walking, balance, health-related quality of life, and patient-reported recovery

Xie et al., 2018 [32]	250 participants from 10 community health centers (5 per arm) were selected and randomly allocated into Tai Chi Yunshou exercise group (TC group) or a balance rehabilitation training group (control group) in an equal ratio	Participants in the TC group received Tai Chi Yunshou exercise training five times per week for 12 weeks and those in control group received balance rehabilitation training five times per week for 12 weeks	A 12-week Tai Chi Yunshou intervention was more effective in motor function, fear of falling and depression than balance rehabilitation training. Tai Chi Yunshou and balance rehabilitation training led to improved balance ability and functional mobility, and both are suitable community-based programs that may benefit for stroke recovery and community reintegration

Zhu et al., 2016 [27]	28 participants with impairments in walking and controlling balance more than six months poststroke were randomly assigned to a land-based therapy (control group, *n* = 14) or hydrotherapy (study group, *n* = 14)	Participants underwent individual sessions for four weeks, five days a week, for 45 minutes per session	The Berg balance scale, functional reach test, 2-minute walk test, and the timed up and go test scores had improved significantly in each group (*p* < 0.05). The mean improvement of the functional reach test and 2-minute walk test were significantly higher in the aquatic group than in the control group (*p* < 0.01). A relatively short program (four weeks) of hydrotherapy exercise resulted in a large improvement in a small group (*n* = 14) of individuals with relatively high balance and walking function following a stroke

The article "Identification of Good Practices in Long-Term Exercise-Based Rehabilitation Programs in Stroke Patients" was published in 2021. Journal: Biomed Res Int.

**Table 2:** Overview of the 10 partners' exercise-based interventions after stroke.

Intervention/type/country	Participants	Intervention	Main findings
Stationary vs. home rehabilitation/study/Croatia [16]	Intervention group size 60 hemorrhagic and ischemic stroke patients (30 in stationary rehabilitation, 30 in home rehabilitation)	Stationary rehabilitation: kinesitherapy, electrotherapy, hydrotherapy, medical care and thermal pools, during 3 weeks. Rehabilitation at home: physiotherapy, individual exercises, stretching, joint mobilization, and massages	Stationary rehabilitation is superior in quality of life improvement, total functional outcome, improvement of the upper limb and balance. Comorbidities are better regulated in patients in stationary rehabilitation

Rehabilitation with mirror-induced visual illusion/study/Croatia [17]	31 ischemic and hemorrhagic stroke patients with both right and left hemiparesis (experimental group: 17)	Experimental group: standard rehabilitation treatment with additional mirror therapy, once a day, 5 days per week for 15 minutes per day, exercises divided into three series of 5 minutes; control group: standard rehabilitation treatment	Mirror therapy improved motor function in the upper limb, leading to a greater potential of self-care and activities of daily living

Robotic rehabilitation/study/Czech Republic [18]	38 stroke patients (20 experimental group, 18 control group)	Physiotherapy for 5 hours weekly and ergotherapy 2.5 hour weekly	Diminution of spasticity (MAS median form 2 to 1 in the experimental group versus 2 to 1+ in the control group) and an improvement in the hand grip functions

Amadeo instrument in chronic rehabilitation/Study/Czech Republic [19]	12 hemorragic and ischemic stroke patients	Stretching of the spastic muscles of the upper acre extremities followed by intense training using an Amadeo instrument for 45 minutes. The first 5-20 minutes were devoted to the passive exercises (CPM and CPMplus), which alternated with assisted exercise, then active training—games balloon, firefighter, recycling, apple picker, shootout (one month, three times weekly)	No statistically significant improvement on motor functions of upper extremity, hand grip strength, motion range of fingers

Cervical isometric exercises/Study/Greece [20]	37 stroke patients with hemiparesis and symptoms of dysphagia	Standard physical and speech therapy plus cervical isometric exercises carried out in all 4 directions, four repetitions for 10 minutes three times a day for 12 consecutive weeks	Patients improved cervical alignment, in both coronal and sagittal plane and deglutition

Exercise rehabilitation program with experiential music/Study/Greece [21]	24 ischemic and hemorrhagic stroke patients	Patients followed a 6 months music-based exercise program, at a frequency of 4 training sessions per week, for 45 minutes each session. Each training session included group activities supported by experiential/traditional music throughout each lesson, with a 5 minutes warm-up period of breathing and flexibility exercises followed by the main part of upper and lower body strengthening, balance and co-ordination exercises on sitting and standing position and trunk movements performed at a moderate intensity and a cool-down period of 5-10 minutes of patients holding hands while moving slowly in a circle listening to music	Recovery rate (defined as the improvement of cognitive and motor skills of the limb in the affected site, with an increase of muscle strength at least by 1/5 and with emotional progress) was higher when exercise rehabilitation program was accompanied by an enriched sound environment with experiential music on stroke patients

Adaptive physical activity with therapeutic patient education/study/Italy [22]	229 ischemic and hemorrhagic stroke patients	Three group sessions of interactive therapeutic patient education (TPE) and 8 weeks of twice weekly adaptive physical activities (APA) exercise sessions have been delivered. Duration: 60 minutes. Intensity of training: progressively increased	APA associated to TPE results to be a useful and potentially cost-effective intervention to maintain and improve activities of daily living, reduce fractures and recourse to rehabilitation treatments. It has been observed a significant improvement on mobility, balance, and on patients' perception of recovery from the acute phase

Low-intensity endurance and resistance training/Study/Italy [23]	35 ischemic and hemorrhagic stroke patients	8-week program composed of an endurance phase based on walking training (weeks 1-4) followed by a mixed phase (weeks 5-8) mainly focusing on muscle-strength training. Frequency: 3 sessions/week. Duration: 60 minutes. Intensity of training: progressively increased	Improvement of mobility, lower-limb strength and power, balance, gait speed, and quality of life

Virtual reality and traditional physiotherapy/action/Lithuania (unpublished)	8 ischemic stroke patients	Individualized computer programs of movement training exercises. Program length: 4 weeks. Frequency: 2 sessions/week. Duration: 30 minutes	Positive influence on patients' balance and coordination (ataxy). Strengthened patients' motivation

Gait training with KinisiForo system/action/Lithuania (unpublished)	12 stroke patients	Gait training with KinisiForo system (3 weeks)	Improvements in trunk control, gait symmetry, and walking speed

The article "Identification of Good Practices in Long-Term Exercise-Based Rehabilitation Programs in Stroke Patients" was published in 2021. Journal: Biomed Res Int.

**Table 3:** The main characteristics of the strategies collected from the partners' countries' interventions.

Action type	Usage
Education/data collection about stroke rehabilitation benefits	There are still many patients (and even healthcare professionals) who are not totally convinced about the benefits of a long-term stroke rehabilitation program. Before trying to improve participation rates, there must be a consensus between the necessity and importance of long-term stroke rehabilitation. Promotional studies are essential.

Test new methodologies to overcome barriers	Mitigation of the barriers to participation is necessary. The number of studies involving large patient cohorts and a long timeframe is still extremely limited. Scientific studies are needed to identify ways to overcome the main causes of non-participation. Countries with more developed stroke rehabilitation system need to focus on the involvement of the hard to reach populations and therefore design specialized studies.

Identify exercise training variables	MY WAY project's golden rules need to identify the main training variables (intensity, frequency, duration, and type of exercise) that could lead to efficient exercise-based stroke rehabilitation. Countries with more developed stroke rehabilitation system need to aim the implementation of safe and effective exercise training programs and therefore design specialized studies.

Implement methodologies to increase participation	The lack of evidence in support of new technologies means that very few ideas have been implemented on a large scale, and consequently, long-term stroke rehabilitation participation rates have not improved significantly. Increasing participation need not necessarily rest on the evidence of rigorous controlled trials. Many centers/countries are using more of the traditional methods to achieve better results.

The article "Identification of Good Practices in Long-Term Exercise-Based Rehabilitation Programs in Stroke Patients" was published in 2021. Journal: Biomed Res Int.

## Data Availability

Data is available on request.
